This article has been retracted.

# Transgenic mice overexpressing the ALS-linked protein Matrin 3 develop a profound muscle phenotype

**DOI:** 10.1186/s40478-016-0393-5

**Published:** 2016-11-18

**Authors:** Christina Moloney, Sruti Rayaprolu, John Howard, Susan Fromholt, Hilda Brown, Matt Collins, Mariela Cabrera, Colin Duffy, Zoe Siemienski, Dave Miller, Maurice S. Swanson, Lucia Notterpek, David R. Borchelt, Jada Lewis

**Affiliations:** 1 Center for Translational Research in Neurodegenerative Disease, University of Florida, Gainesville, FL USA; 2 Department of Neuroscience, University of Florida, Gainesville, FL USA; 3 Department of Molecular Genetics and Microbiology, Center for NeuroGenetics and the Genetics Institute, University of Florida, College of Medicine, Gainesville, FL USA; 4 McKnight Brain Institute, Department of Neuroscience, University of Florida, Gainesville, FL USA

**Keywords:** Matrin 3, Transgenic mouse model, ALS, Distal myopathy

## Abstract

Amyotrophic lateral sclerosis (ALS) is a progressive neurodegenerative disorder of upper and lower motor neurons. Mutations in the gene encoding the nuclear matrix protein Matrin 3 have been found in familial cases of ALS, as well as autosomal dominant distal myopathy with vocal cord and pharyngeal weakness. We previously found that spinal cord and muscle, organs involved in either ALS or distal myopathy, have relatively lower levels of Matrin 3 compared to the brain and other peripheral organs in the murine system. This suggests that these organs may be vulnerable to any changes in Matrin 3. In order to determine the role of Matrin 3 in these diseases, we created a transgenic mouse model for human wild-type Matrin 3 using the mouse prion promoter (MoPrP) on a FVB background.

We identified three founder transgenic lines that produced offspring in which mice developed either hindlimb paresis or paralysis with hindlimb and forelimb muscle atrophy. Muscles of affected mice showed a striking increase in nuclear Matrin 3, as well as the presence of rounded fibers, vacuoles, nuclear chains, and subsarcolemmal nuclei. Immunoblot analysis of the gastrocnemius muscle from phenotypic mice showed increased levels of Matrin 3 products migrating at approximately 120 (doublet), 90, 70, and 55 kDa. While there was no significant change in the levels of Matrin 3 in the spinal cord in the phenotypic mice, the ventral horn contained individual cells with cytoplasmic redistribution of Matrin 3, as well as gliosis. The phenotypes of these mice indicate that dysregulation of Matrin 3 levels is deleterious to neuromuscular function.

**Electronic supplementary material:**

The online version of this article (doi:10.1186/s40478-016-0393-5) contains supplementary material, which is available to authorized users.

## Introduction

Amyotrophic lateral sclerosis (ALS) is a degenerative disorder of upper and lower motor neurons, and is characterized by progressive paralysis, typically leading to death three to five years following diagnosis due to respiratory failure [25]. Lower motor neuron degeneration results in muscle atrophy and weakness, as well as fasciculations. Upper motor neuron degeneration results in spasticity, and increased reflex activity, along with clonus, Hoffmann sign, and Babinski sign [25]. Initial symptoms are typically weakness in hands or legs, and can include dysphagia and slurred speech [25]. Age, family history, and even some evidence of possible environmental factors can all serve as risk factors for ALS [25]. Pathological features of ALS include atrophy of motor neurons with astrocyte and microglia activation [19]. Abnormal protein aggregation or localization within neurons and glia can also be observed, with the specific protein involved varying depending on the cause [25]. There is no effective treatment for this disease and currently the only treatment, riluzole, merely slows the progression of the disease and prolongs lifespan by 3 months [25].

The recent growth in our knowledge about the genetic underpinnings of ALS could provide new opportunities for therapeutic target identification and subsequent development of therapies. Most patients with ALS report no known family history of the disease and are classified as sporadic ALS; whereas, about 10% of cases are classified as familial with Mendelian patterns of inheritance. Interestingly, about 10% of sporadic ALS cases turn out to have mutations in genes associated with familial disease. The gene mutations for about one third of familial ALS cases remain unknown [22]. Over 20 years ago, mutations in superoxide dismutase 1 (*SOD1*) were identified as causative for ALS [24]; however, the recent wave of genetic discoveries in the field has implicated genes such as TAR DNA-binding protein (*TARDBP*) [28], fused in sarcoma (*FUS*) [13, 29], and the G_4_C_2_ repeat expansion in chromosome 9 open reading frame 72 (*C9orf72*) [5, 23]. More recently, Johnson and colleagues used exome sequencing to identify three coding mutations (Phe115Cys, Thr622Ala, and Pro154Ser) in Matrin 3 (*MATR3* gene; MATR3 protein) in both familial and sporadic ALS [12]. Individuals with the Phe115Cys mutation died from respiratory failure within 5 years of symptom onset, consistent with the typical course of ALS. Immunohistochemistry revealed strong nuclear and variable cytoplasmic staining of Matrin 3 in the spinal cord [12]. Another mutation, Ser85Cys, was originally identified as a cause of distal myopathy in a large American family [27]; however, upon discovery of a link between mutant Matrin 3 and ALS, this family was re-evaluated and reclassified to slowly progressive ALS [12]. In contrast, Müller and colleagues reported 16 patients with distal myopathy harboring the same Ser85Cys Matrin 3 mutation that lacked lower motor neuron involvement that is typically seen in ALS [16].

Distal myopathy is a group of disorders in which weakness and atrophy of the upper and lower distal muscles, such as muscles in the hands and feet, are initial manifestations of the disease. In 1998, Feit and colleagues described affected individuals of a Caucasian, Tennessean family having a novel vocal cord and pharyngeal weakness with autosomal dominant distal myopathy, and localized the gene to chromosome 5q31 using genome screening and DNA-pooling [6]. This family had an average age of onset at 45.7 years, ranging from 35 to 57 years, with initial presentations usually being ankle dorsiflexion weakness and foot drop. Muscle biopsies from affected individuals showed rimmed vacuoles, as well as atrophic fibers consistent with denervation, and electromyogram and nerve conduction studies pointed towards a myopathy in some but not all individuals examined [6]. Electron microscopy studies showed no inclusions or amyloid deposits [6]. Senderek and colleagues later discovered the missense Ser85Cys mutation in Matrin 3 to be the cause of disease in this family [27]. Additionally, a Bulgarian and an Asian kindred have been found to have this mutation in association with distal myopathy [27, 34].

Matrin 3 is a highly conserved, slightly acidic nuclear matrix protein of 125 kDa [17]. It has two RNA recognition motifs in tandem, two zinc finger domains, a nuclear localization signal, a nuclear export signal, and a membrane retention signal [10]. Matrin 3 has roles in retention of hyper-edited RNA to the nucleus [35], DNA repair due to double strand breaks [26], alternative splicing [4], and even neuronal death due to NMDA-receptor activation [8]. We have previously shown that disease-causing mutations in Matrin 3 do not strikingly alter normal nuclear localization of the protein, nor does the protein form inclusions in H4 neuroglioma and Chinese Hamster Ovary cells [7]. There is minimal knowledge of the normal function of Matrin 3 in spinal cord and the muscle. The mechanism underlying the pleomorphic nature of Matrin 3 mutations is entirely unknown. We recently characterized endogenous Matrin 3 expression throughout the development and aging of the postnatal mouse in the CNS and periphery. We found that, in the brain and spinal cord, Matrin 3 levels were higher in earlier stages of development, and decreased as the mouse ages. Interestingly, the muscle and spinal cord, organs that are involved in either ALS or distal myopathy, have relatively low levels of Matrin 3 compared to the brain and other organs in the periphery. This finding could suggest that these organs may be vulnerable to any changes in Matrin 3 function [21]. Humans with congenital chromosomal translocations that disrupt the 3′ untranslated region (UTR) of Matrin 3 mRNA have developmental heart defects [20]. In 2015, Quintero-Rivera and colleagues created a knockout model, finding homozygous null mice die in early embryogenesis [20]. Heterozygous knockout mice showed abnormalities in the heart, similar to those seen in humans with the translocation altering the 3′ UTR of Matrin 3; however, no ALS or distal myopathy phenotypes were reported. Since there was no significant change in Matrin 3 expression between heterozygous knockout and wild-type mice the link of Matrin 3 to the reported phenotype is unclear [20]. In an effort to provide critical tools for understanding the role(s) of Matrin 3 in normal and, potentially, disease biology, we have created multiple lines of transgenic (Tg) mice expressing human wild-type Matrin 3. These Tg mice develop an incompletely-penetrant phenotype that includes hindlimb paresis or paralysis, as well as hindlimb and forelimb muscle atrophy, indicating that the function of Matrin 3 has a direct impact on neuromuscular function.

## Materials and methods

### Animal husbandry

Mice were kept on a 12 h light/12 h dark cycle with ad libitum access to food and water. All procedures were approved by the Institutional Animal Care and Use Committee of the University of Florida, and complied with the National Institute of Health’s “Guide for the Care and Use of Laboratory Animals.”

### Generation of transgenic animals

To generate wild-type human *MATR3* mice, human *MATR3* cDNA in the pCMV-Sport6 clone (ThermoScientific #MHS6278-202757255) was cloned into the *Sal* I site of a modified pEF-BOS vector using the InFusion HD cloning kit, (Clontech, catalog #639649). Then this human *MATR3* vector was digested with *Sal* I, gel purified, and the cDNA ligated into the *Xho* I site of the MoPrP vector [2]. The transgene was microinjected into FVB/NJ fertilized oocytes (Jackson Laboratory), and implanted into pseudopregnant females. Five founders were mated with FVB/NCr (Charles River) to generate F1 offspring. Tg mice were identified by PCR using primers: (PrP-Sense) 5′GGGACTATGTGGACTGATGTCGG, (PrP-Antisense) 5′CCAAGC CTAGACCACGAGAATGC, (endogenous *MATR3*) 5′AGCAAGAGCTTGGACGTGTG.

### Phenotyping of animals

Animals were classified into two phenotypic stages: mild to moderate (MM) and severe (S). Although there was not a significant difference of body weight of the MM mice versus non-transgenic (NT) mice, a trained observer cognizant of genotype used a combination of initial motor deficits, body size and muscle size to identify the subset of transgene positive animals that were categorized as mildly phenotypic. In contrast, members of the UF Animal Care Services who were blinded to genotype used the presentation of hindlimb paralysis or paresis to determine if the animals had reached end point which we classified as severe phenotype.

### Harvesting

Mice were euthanized either by cervical dislocation or anesthetized with isoflurane and euthanized by exsanguination with phosphate buffered saline (PBS) perfusion. The brain was hemisectioned down the sagittal midline, with half immersion fixed (10% formalin) and the other half frozen on dry ice. The spinal column, hindlimb, and forelimb were dissected and immersion fixed in 10% formalin. After 24 h, fixed brain, hindlimb and forelimb were transferred into PBS while the spinal cord was extracted from the spinal column, and fixed for another 24 h prior to transferring to PBS. All the tissues were stored in PBS at 4 °C until processing. The cervical portion of the spinal cord, and hindlimb and forelimb muscles were snap frozen on dry ice and stored at -80 °C until lysate preparation.

### Lysate Preparation

Frozen tissue was homogenized in six volumes of the weight in homogenization buffer [50 mM Tris pH7.5, 300 mM NaCl, 5 mM EDTA, 1% Triton, 1x protease inhibitor (Sigma, catalog # 8340), 1x phosphatase inhibitor #1 (Sigma, catalog # P0044), 1x phosphatase inhibitor #2 (Sigma, catalog # P5726)], which was then stored in aliquots at −80 °C. An aliquot was further diluted to ten volumes of homogenization buffer. The samples were sonicated, and SDS was added to a final concentration of 2%. The samples were centrifuged for 20 min at 4 °C at 40,000 rpm. The supernatant was collected and protein concentration was determined using BCA protein assay (Pierce, Rockford, IL).

### Western blotting

For Coomassie blue staining, equal amounts of protein were resolved on a 4–20% Tris-glycine gel. The gel was stained with Coomassie blue for 2 h, destained overnight, and imaged on the InGenius 3 using the GeneSys software (SynGene). For immunoblotting, equal amounts of protein were resolved on a 3–8% Tris-acetate gel and transferred onto a nitrocellulose membrane for 90 min at 200 mA. The blots were blocked in 5% milk in Tris-buffered saline (TBS) for an hour and were incubated overnight with rabbit α-Matrin 3 antibody (1:10,000, Novus Biologicals, catalog # NB100-1761) or mouse α-GAPDH antibody (1:5,000, Meridian Life Sciences, catalog # H86504M) diluted in 5% milk/TBS. Following washes in TBS, the blots were incubated with horseradish peroxidase-conjugated α-rabbit or α-mouse for 1 h (1:5,000, Jackson ImmunoResearch Laboratories, Inc., rabbit catalog # 711-036-125, mouse catalog # 715-036-150). Following washes in TBS, membranes were incubated with ECL-Plus reagent (Fisher, catalog # 509049326) and imaged on PXi using the GeneSys software (SynGene).

### Immunohistochemistry

The spinal cord, gastrocnemius from the hindlimb, and bicep from the forelimb were paraffin embedded and sectioned into 5 μm sections. Following deparaffinization, sections were steamed in 10 mM citrate with 0.05% Tween-20 for 30 min (Matrin 3, GFAP) or incubated in 70% formic acid for 10 min (Iba-1). Following alternating washes in water and PBS, sections were blocked in 0.3% H_2_O_2_/PBS for 20 min. After thorough washes in Milli-Q H_2_O, sections were blocked with 10% normal goat serum (Vector Labs, catalog # S1000) in PBS and 0.05% Tween-20 (PBS-T) for 30 min at room temperature. Sections were then incubated with rabbit α-Matrin 3 antibody (1:1,000,Novus Biologicals, catalog # NB100-1761), rabbit α-Iba1 (1:500, Wako Chemicals USA, catalog # NC9288364), or rabbit α-GFAP (1:1,000, Dako, catalog # Z0334) in 5% normal goat serum/PBS-T overnight at 4 °C. Subsequently, the sections were rinsed with PBS-T and incubated with biotinylated α-rabbit antibody (1:500, Vector Labs, catalog # BA1000) in 5% normal goat serum/PBS-T for 30 min at room temperature. The signal was detected with a standard peroxidase ABC system (Vector Labs, catalog # PK6100) with DAB as the chromogen, counterstained with hematoxylin, dehydrated and cover-slipped using Cytoseal (Thermo Scientific, catalog #8310-4).

### Neuromuscular junction analysis

For immunofluorescence, 4 Tg and 4 NT were euthanized by cervical dislocation. The Tg mice presented with a MM phenotype. The Tg mice were 10.1 and 7.3 months of age, NT mice were ~10 months and 7.3 months. Diaphragm and gastrocnemius (1/4^th^ cut longitudinally) were dissected, and fixed in 4% paraformaldehyde for 10 min. After three 5 min washes in PBS, muscles were permeabilized for 30 min in 2% TritonX-100 in PBS. Muscles were then blocked overnight at 4 °C in blocking solution (1% TritonX-100, 4% BSA in PBS) and followed by incubation with mouse α-synaptotagmin (1:200, Zebrafish International Resource Center, catalog # ANZNP-1) and chicken α-neurofilament heavy polypeptide (1:5,000, EncorBio, catalog # CPCA-NF-H) antibodies diluted in blocking solution for 24 h at 4 °C. Muscles were washed six times for 30 min each in PBS and incubated in anti-mouse Alexa 488 (1:200, Invitrogen, catalog # A21200), anti-chicken Alexa 647 (1:1,000, LifeTechnologies, catalog # A21449), and Alexa 597 Bungarotoxin (1:1,000, LifeTechnologies, catalog # B13423), diluted in blocking solution for 24 h at 4 °C. After washing six times for 30 mins in PBS, muscles were mounted with VECTASHIELD anti-fade mounting medium with DAPI (Vector Labs, catalog #H-1200).

### Confocal microscopy

Images were captured using the Nikon A1RMPsi-STORM4.0 (Alexa 594, emission wavelength 595 nm; Alexa 647, emission wavelength 700 nm, DAPI, emission wavelength 450 nm; Alexa 488, emission wavelength 525 nm). Images for neuromuscular junctions were acquired using a z-stack of 2 μm thick slice sections throughout the muscle.

### Statistical analysis

Statistical analysis of the body weights between NT controls and Tg mice was performed with an unpaired, Student’s t test using GraphPad Prism version 6.00 (GraphPad Software) and *P* ≤ 0.05 was considered to be statistically significant.

## Results

We generated Tg mice using the MoPrP promoter to drive expression of full length, wild-type human Matrin 3. All five founders we initially identified (1579, 1576, 1573, 72, 70) transmitted the transgene, and we identified four of these Tg founder lines (1579, 1576, 1573, 72) that overexpressed Matrin 3 in the gastrocnemius, compared to NT littermates. To date, three of these founder lines (1579, 1576, and 1573) have produced offspring that developed a phenotype of hindlimb paresis or paralysis (Fig. 1a; Table 1) that is strikingly different from the normal phenotype observed in NT mice (Fig. 1b). Founder line 1579, which appeared to be a mosaic, produced six phenotypic F1 Tg mice (5 males and 1 female) and eight asymptomatic F1 Tg mice. These mice developed a phenotype at a mean age of 1.2 months, with a range from 0.9 to 1.4 months. Since these phenotypic mice reached endpoint before breeding age, we were unable to establish a continuous breeding line of phenotypic mice from this founder. Gross observation of the limbs of paralyzed mice from founder line 1579 showed overall hindlimb (Fig. 1c, arrows) and forelimb (Fig. 1e, asterisks) muscle atrophy compared to NT littermates (Fig. 1d, f).

**Fig. 1:** Phenotype of transgenic mice from Fo. 1579 (age of onset ~1.4 months [m]). **a** Tail hang of Tg mouse compared to **b** NT mouse. **c** Hindlimb muscle atrophy of Tg mouse compared to **d** NT mouse. **e** Forelimb muscle atrophy of Tg mouse compared to **f** NT mouse. *Arrow* indicates gastrocnemius. * indicates triceps

**Table 1:** Tg and NT mice used in the study. Founder line, gender, genotype, age at harvest, stage of phenotype, and body weight is reported

Founder Line	Animal ID	Gender	Genotype	Age at harvest (m)	Stage	Body Weight (g)
1579	MA22.7	M	Tg	0.9	S	13.2
	MA83.1	F	Tg	1.1	S	10.8
	MA13.8	M	Tg	1.3	S	16.9
	MA35.8	M	Tg	1.3	S	15.0
	MA1.4	M	Tg	1.4	S	13.5
	MA7.8	M	Tg	1.4	S	16.6
1576	MA39.3	M	Tg	4.1	S	20.1
	1576	F	Tg	4.8	S	21.8
	MA75.2	F	Tg	10.1	MM	27.3
	MA75.3	F	Tg	10.1	MM	20.1
	MA75.4	F	Tg	10.1	MM	27.2
	MA39.1	F	Tg	10.5	S	17.7
1573	MA95.3	F	Tg	7.3	MM	19.9
	MA16.2	M	Tg	8.4	S	16.6
	MA2.7	M	Tg	9.2	S	20.1
	MA16.1	F	Tg	13.8	S	16.9
Control	MA83.2	F	NT	1.1		20.1
	MA1.5	M	NT	1.4		25.2
	MA7.6	M	NT	1.5		23.2
	MA1.1	F	NT	1.6		20.8
	MA13.6	M	NT	1.6		21.9
	MA35.7	M	NT	2		26.0
	1578	F	NT	4.8		20.5
	F77.3	F	NT	7.3		25.8
	MA16.4	M	NT	8.6		39.4
	F36.1	F	NT	9.7		24.7
	F58.5	F	NT	10		29.5
	F58.6	F	NT	10		28.0
	MA75.1	F	NT	10.1		31.6

*m* months, *S* severe phenotype, *MM* mild to moderate phenotype

Founder 1576 developed decreased hindlimb muscle size and dystocia at 4.8 months which required euthanasia. Two F2 Tg offspring from this founder line were classified as severely affected and developed paralysis and hindlimb muscle atrophy; a male at 4.1 months and a female at 10.5 months. An additional three F3 female Tg mice from Line 1576 were classified as mild to moderately affected at 10.1 months.

One F1 Tg male and one F2 Tg male offspring from founder line 1573 became phenotypic at 9.2 and 8.4 months, respectively, both exhibiting hindlimb muscle atrophy. The latter had an abnormal tail hang and exhibited very little movement when encouraged to walk. A F2 Tg female from this line exhibited muscle atrophy and paresis at ~12 months, and was euthanized at 13.8 months. An additional female F3 Tg mouse from this founder line was analyzed with a mild to moderate phenotype at 7.3 months. The founder line of origin, sex, age at analysis, phenotype at euthanasia, and body weight for each experimental animals is detailed in Table 1.

In addition to the profound motor phenotype that developed in these mice, there was a striking and significant difference in body weights between age-matched NT controls (Mean +/- Std Dev; 22.9 +/- 2.4 g) and Tg mice (14.3 +/- 2.3 g) that were classified as severely affected within founder line 1579 (student’s t-test, *p* < 0.0001; Table 1). Similarly, there was a significant difference (student’s t-test, p = 0.0033) in body weight between age-matched NT control mice (28.5 +/- 6 g) and severely affected Tg mice (18.9 +/- 2.1) from founder lines 1573 and 1576 (combined). Because of the limited number of mice that have been analyzed at the MM phenotypic stage, similar comparisons were not made.

All phenotypic Tg mice, regardless of founder of origin, had striking and similar pathology in the gastrocnemius muscle, which included rounded muscle fibers of variable size (Fig. 2a, asterisks) and an increase in subsarcolemmal nuclei (Fig. 2a, arrowheads). Another feature of the gastrocnemius of the Tg mice was the presence of subsarcolemmal vacuoles (Fig. 2a, inset). In addition to the increased size of nuclei in the Tg mice (Fig. 2a-b) compared to the NT mice (Fig. 2c-d), there were a few instances of nuclear chains seen in longitudinal sections of the muscle (Fig. 2b, arrow) of phenotypic Tg mice. There was an increase in nuclear Matrin 3 immunostaining in the muscle of Tg mice (Fig. 2e-f) compared to the NT mice (Fig. 2g-h), although expression was heterogeneous throughout the muscle, even in nuclear chains (Fig. 2f, inset). Matrin 3 immunostaining in the cytoplasm was also present in the Tg mice, but was a rare occurrence (Fig. 2e, inset). These findings were not exclusive to the gastrocnemius muscle, as they were also seen in the forelimb (Additional file 1: Figure S1). Qualitatively, the pathology observed in the hindlimbs was more severe than that observed in the forelimbs. The gastrocnemius from three 10 months female mice from founder line 1576 and one 7.3 month female mouse from founder line 1573, each of which displayed a MM phenotype, were analyzed for neuromuscular junction (NMJ) abnormalities in comparison to age matched NT mice. The gastrocnemius was double labeled for synaptotagmin 2 (ZNP1) and α-bungarotoxin (BTX) to visualize the pre-synaptic terminals and acetylcholine receptors on the muscle fibers, respectively. The NMJs were profoundly altered in the Tg muscle compared to the NMJ in NT muscle. The Tg NMJs have a collapsed morphology as detected by the loss of the classic pretzel shaped BTX labeling, decrease in overall post-synaptic junction size, and the presence of fragmentation (Fig. 3, arrowheads). We also observed a pronounced reduction in overlap between the presynaptic ZNP1 and postsynaptic BTX in the Tg muscle, as compared to NT muscle.

**Fig. 2:** Striking muscle pathology of gastrocnemius in Tg mice from Fo. 1579. **a** Transverse and **b** longitudinal sections from phenotypic Tg mouse stained with H&E compared to **c** transverse and **d** longitudinal of NT mouse. **e** Matrin 3 immunohistochemistry of transverse and **f** longitudinal sections from phenotypic Tg show an increase in Matrin 3 immunoreactivity compared to NT **g** transverse and **h** longitudinal sections. * indicates rounded fiber. *Arrow head* indicates subsarcolemmal nucleus. *Arrow* indicates nuclear chain. Scale bars measure 25 μm

**Fig. 3:** NMJs of MM Tg mice have structural abnormalities compared to NT mice from Fo. 1576 at ~10 m of age. α-bungarotoxin (BTX), synaptotagmin (ZNP1) were used to label the NMJs, with BTX identifying post-synaptic acetylcholine receptor clusters and ZNP1 visualizing the pre-synaptic nerve terminal. Arrowheads indicate fragmented NMJs. Scale bar measures 100 μm

Spinal cords showed instances of cytoplasmic redistribution of Matrin 3 with puncta in neurons of the ventral horn in the phenotypic Tg mice (Fig. 4a, inset) compared to Matrin 3 distribution in NT mice. Additionally, we observed qualitatively stronger nuclear immunoreactivity of Matrin 3 in the spinal cords of Tg mice than in the NT mice; however, this was not uniform across all Tg mice (Fig. 4a-b). Iba-1 positive microglia (Fig. 4c-d) and GFAP positive astrocytes (Fig. 4e-f) revealed prominent gliosis in the ventral horn of the spinal cord of phenotypic Tg Matrin 3 mice, while NT spinal cords showed minimal immunostaining. In some cases, the neurons with high levels of cytoplasmic Matrin 3 were surrounded by glia (Fig. 4g, arrow).

**Fig. 4:** Cytoplasmic Matrin 3 re-localization and gliosis in ventral horn of the spinal cord in phenotypic Tg mice. **a** Matrin 3 immunohistochemistry shows cytoplasmic redistribution in the Tg (Fo. 1579) ventral horn compared to **b** NT mice. **c** Iba-1 immunohistochemistry shows microgliosis in Tg (Fo. 1579) mice compared to **d** NT mice. **e** GFAP immunohistochemistry shows increase staining indicative of astrocytosis in Tg (Fo. 1579) mice compared to **f** NT mice. **g** Neuron with cytoplasmic re-localization of Matrin 3 in the ventral horn of the spinal cord, surrounded by glia, as indicated by the arrow, from phenotypic founder 1576. Scale bars measure 25 μm

In preparation for immunoblot analysis, we used Coomassie blue staining of SDS-soluble fractions of the gastrocnemius to assess protein content in our tissue homogenates. Interestingly, the phenotypic Tg mice from founder line 1579 showed a different banding pattern compared to NT mice, including a dramatic reduction of a high molecular weight band above 170 kDa in the Tg versus the NT mice (Fig. 5a). The size of this band is consistent with the myosin heavy chain. In the Tg mice from founder line 1579, there was also a striking increase in a band migrating at ~70 kDa compared to age matched NT mice (Fig. 5a). Western blots of the muscle showed that the phenotypic Tg mice contained multiple bands that were immunopositive for Matrin 3 at approximately 120 (doublet), 90, 70, and 58 kDa that were barely detectable in NT mice (Fig. 5b). As observed in the Coomassie staining, the banding profile of the muscle homogenate from phenotypic Tg mice derived from founder line 1579 was generally different than that observed in phenotypic Tg mice from founder lines 1576 or 1573 when immunostained with a Matrin 3 antibody. Additionally, there is a strong Matrin 3 immunopositive band at ~70 kDa in the phenotypic founder line 1579 Tg mice, potentially explaining the presence of a strong 70 kDa band in the Coomassie stained gel for those mice (Fig. 5b).

**Fig. 5:** Biochemical analysis of SDS-soluble fraction of the gastrocnemius. **a** Coomassie stain of homogenate (25 μg protein) for Fo. 1579, 1576, and 1573. Average age for indicated group is reported months (m). All Tg mice had similar phenotypes at the age analyzed. Tg mice with a phenotype from line 1579 have a striking change in protein banding pattern compared to NT mice including a nearly complete loss of high MW (~170 kDa) band which may represent Myosin Heavy Chain. In contrast, banding pattern for phenotypic Tg mice from lines 1576 and 1573 were similar to NT mice on the Coomassie-stained gel. **b** Matrin 3 immunoblotting (15 μg protein) from NT and phenotypic Tg mice shown in Coomassie blot (a) shows the consistent presence of lower molecular weight bands in affected 1579 mice. **c** Matrin 3 immunoblotting (20 μg protein) from non-phenotypic, Tg mice (~2 m of age) from Fo. 1576 and 1573 show lower molecular weight bands similar that that observed in phenotypic mice from line 1579. *Bottom panel* is GAPDH as a loading control. * indicates homogenate from phenotypic Fo. 1576 age ~5 m was used as a reference sample. *Arrow head* indicates major Matrin 3 product ~120 kDa that often runs as a doublet

We could not explain the disparity between observed Matrin 3 immunopositive protein bands in the Tg mice from founder line 1579 versus 1576 and 1573; however, we suspected that the young age at which mice from founder line 1579 became phenotypic could underlie this difference. To address this, we analyzed non-phenotypic Tg mice at ~2 months of age from both founder lines 1576 and 1573 (Fig. 5c) against phenotypic Tg mice from founder line 1576 at ~5 months of age (Fig. 5c *Tg). To our surprise, each of the lower molecular weight products observed in the young phenotypic Tg mice from founder line 1579 were also found in the young non-phenotypic Tg mice from founder lines 1576 and 1573. This result suggested that the presence of these lower molecular weight products is most likely reflective of age and not phenotype. In contrast to our data from the muscle of our phenotypic Matrin 3 Tg mice, the brains and spinal cords showed no robust difference of Matrin 3 levels between the phenotypic Tg and NT mice of each line (data not shown). Similarly, there was no striking difference in Matrin 3 levels in the spinal cord between non-phenotypic Tg mice and NT mice, regardless of line (data not shown).

## Discussion

We generated four transmitting, independent lines of novel Tg mice harboring a vector to express full length human Matrin 3. A subset of transgenic mice from three of these lines developed similar gross muscle atrophy and paresis that primarily affected the hindlimbs. Immunohistochemical studies on the gastrocnemius muscle of phenotypic Tg mice, regardless of line, showed rounded and misshapen muscle fibers that were reduced in size, increased and displaced subsarcolemmal nuclei, vacuoles, and variable presence of nuclear chains. Similar pathology was observed in the forelimbs of phenotypic Tg mice, though qualitatively less severe. We observed both astrocytosis and microgliosis in the ventral horn of the spinal cords of affected mice. Additionally, we observed Matrin 3 re-localization in a small subset of neurons within the same region.

Given the presence of pathology in both the muscle and spinal cord of affected mice, we sought to determine if both muscle and spinal cord expressed the transgene. The hindlimbs from phenotypic Tg mice had increased levels of Matrin 3 on the western blot in comparison to NT mice; however, there were no striking differences in Matrin 3 levels in homogenates from total brain and cervical spinal cord between phenotypic Tg mice and NT mice, regardless of founder line. The MoPrP promoter has been repeatedly utilized to efficiently drive expression of FTD/ALS-related and other Tg proteins within the brain and spinal cord [2, 15, 32, 33]; therefore, the lack of overexpression within the CNS was surprising. Since many RNA-binding proteins normally undergo autoregulation to maintain proper levels of mRNA and, subsequently, protein (for review, see [3]), it is possible that there is expression of the human Matrin 3 within the spinal cord and brain, but these tissues are able to efficiently downregulate endogenous expression to maintain normal total levels of Matrin 3. Given the remarkable homology between rodent and human Matrin 3 [1], there is no antibody available to distinguish between the species of origin of the Matrin 3 protein which prevents this inquiry. Alternatively, the Tg expression may not be reflected in global analysis of Matrin 3 levels within the spinal cord; immunohistochemical analysis is suggestive that specific cells have elevated levels of Matrin 3 in the Tg mice. It is possible that localized increases in Matrin 3 levels or function could underlie the changes in the spinal cord of the phenotypic mice that either cause subsequent changes in the muscle or represent an independent, parallel process from that observed in the muscle. Finally, it is possible that pathology first occurs within the muscle, resulting in subsequent changes in motor neurons. This possibility is consistent with the observation that patients carrying the Ser85Cys mutation were initially diagnosed with the distal myopathy and then later ALS [12].

The pathology that we observed in the Matrin 3 Tg mice appears to closely resemble that from distal myopathy cases with Matrin 3 mutation [6, 16, 18, 27, 34]. Many groups have reported gastrocnemius or tibialis anterior muscle containing fibers of variable size, increased subsarcolemmal nuclei, and the presence of vacuoles in affected individuals with Matrin 3 mutations, similar to that observed in our phenotypic mice in the context of wild-type Matrin 3 [6, 16, 18, 27, 34]. The robust increase in Matrin 3 levels within the skeletal muscle of our Tg lines could suggest that any increase in normal levels or function of the protein in the muscle is responsible for the mouse phenotype. Although MoPrP has been previously shown to drive transgenic expression within the skeletal muscle [2], it is surprising that Matrin 3 levels would be driven at higher levels in the muscle compared to the CNS in our lines. It is conceivable that the overexpression of the transgene could overwhelm any existing autoregulatory system in the muscle, allowing for the increase of Matrin 3 levels.

We made an interesting finding during our immunoblotting studies of these mice. In young Tg mice, regardless of line or presence of phenotype, four different bands that were immunopositive with a Matrin 3 antibody were visible. Since we are expressing full length human Matrin 3 from a cDNA construct, these products are not due to alternative splicing of the transgenic mRNA; however, it is possible that these bands originate from alternative splicing of the murine Matrin 3 mRNA that has been induced by expression of the human transgene. Alternatively, it is possible that these bands originate from post-translational modification (cleavage) of either the human or the murine Matrin 3. These bands were only consistently found in young mice, regardless of phenotype. This finding suggests that there may be developmental and/or age-related factors that result in the production of the lower molecular weight bands that are immunopositive for Matrin 3.

In the course of breeding our founder lines, we quickly realized that the founder designated 1579 was likely mosaic. Six of her 14 F1 offspring developed severe paralysis within the first 1.4 months of life; however, this founder remained asymptomatic. Unfortunately, the early phenotype in this line was so severe that we could not establish continuous breeding sublines. The hindlimbs of phenotypic mice from founder line 1579 had high levels of Matrin 3 on western blots; whereas, the asymptomatic Tg mice from this line had Matrin 3 levels equivalent to NT mice (not shown), possibly providing an explanation of incomplete penetrance. We were uncertain as to whether other founders might also be mosaic and we adopted a strategy of breeding multiple F1 offspring from the other founders to determine whether we could identify mice that developed phenotypes at ages more compatible with maintaining breeding lines of mice. From this strategy, we identified two offspring from founder line 1576 and 3 offspring from founder line 1573 that developed the same severe paralytic phenotypes seen in the offspring from founder 1579. Founder 1576 eventually developed dystocia and paresis at 4.8 months of age, but most of her offspring were asymptomatic; whereas, Founder 1573 remained asymptomatic. There were two distinct sublines that arose from founder 1576 – a subline of Tg mice that had levels of Matrin 3 equivalent to the phenotypic founder 1576 and a subline of Tg mice in which Matrin 3 levels were not different from NT (data not shown), suggestive that this founder was also probably mosaic, potentially explaining the partial penetrance of the phenotype. We believe that all of our founder mice may have been mosaic to some degree. We do not yet know whether we will be able to produce a subline from offspring of either of these two founders that exhibits a highly penetrant, reproducible phenotype; however, we (CM) have been able to use a qualitative cage assessment for early stage abnormalities which has thus far tracked with mice that go on to develop pathology. Since these are the first Tg mice to be generated for Matrin 3, and we observed disease-relevant phenotypes, and the phenotypes were observed in offspring from three different founder mice, we believe our findings are informative regarding the potential impact of Matrin 3 expression on neuromuscular function.

The presence of myopathic phenotypes in these mice suggests that Matrin 3 dysregulation contributes to muscle degeneration. However, the observed mislocalization of Matrin 3, and prominent gliosis, in the spinal cord cannot be dismissed. It is also possible that Matrin 3 dysregulation may cause disease that lies within a spectrum of disease from ALS to myopathy, an event that is not without precedent. Valosin-containing protein (*VCP* gene; VCP protein) is a highly conserved protein in the family ATPase associated with various cellular activities including membrane fusion in endoplasmic reticulum and golgi and nuclear envelope, and protein degradation [9, 14, 30]. In 2004, Watts and colleagues reported that mutations in *VCP* caused an inclusion body myopathy associated with Paget disease of bone and frontotemporal dementia (IBMPFD), which affects muscles and brain [31]. Normally, VCP immunostaining is in endomysial vessels, lipofuscin accumulations, and diffusely through the cytoplasm of the muscle fibers. In IBMPFD, immunostaining showed vacuoles and inclusions in the muscle. In 2010, *VCP* was also implicated in four families diagnosed with ALS by Johnson and colleagues [11]. An autopsy showed motor neuron loss of the brainstem and spinal cord, as well as TDP-43 immunostaining that is seen in ALS [11]. These data indicate that VCP plays a role in both ALS and myopathy, similar to what has been proposed for Matrin 3.

Even though our novel Tg mice show some compelling similarities with the human diseases associated with Matrin 3 mutations, the pathology in these mice is caused by wild-type Matrin 3 and is not specific to a mutation. Overexpression of wild-type Matrin 3 has not been reported in association with either ALS or distal myopathy and conclusive evidence that Matrin 3 mutations cause gain-of-function is absent from the literature. Without understanding how mutant Matrin 3 causes disease, it is premature to assert that these mice are good models for the human condition. However, these mice indicate that Matrin 3 levels may be tightly regulated and Tg expression may interfere with this regulation, resulting in defects in neuromuscular function. These new mice may serve as a tool to help bridge our gaps in knowledge regarding Matrin 3 function in the neuromuscular system. If we are able to establish a highly penetrant line of transgenic mice that can be subsequently bred, as it appears we may have now done, these mice will also be a critical resource for comparison to transgenic mice expressing mutant Matrin 3 when they become available so that we can dissect the role that Matrin 3 plays in disease biology. Finally, they will provide a tool which will allow us to study the interaction of Matrin 3 with other key players in neurodegeneration and/or myopathy.

## Conclusion

In summary, we have demonstrated that overexpression of wild-type Matrin 3 induces profound muscle pathology and motor phenotypes in Tg mice.

## Additional file

Additional file 1: Figure S1. Muscle pathology of bicep in phenotypic Tg mice from line 1579. **a** Transverse and **b** longitudinal sections from a phenotypic Tg mouse stained with H&E show multiple pathologies when compared with **c** transverse and **d** longitudinal sections from a NT mouse. **e** Transverse and **f** longitudinal sections from a phenotypic Tg mouse show an increase in Matrin 3 immunoreactivity compared to **g** transverse and **h** longitudinal sections from a NT mouse. * indicates rounded fiber. Arrow head indicates internalized nuclei. Scale bars measure 25 μm. (DOCX 1919 kb)

## Abbreviations

ALS: Amyotrophic lateral sclerosis
BTX: α-bungarotoxin
*C9orf72*: Chromosome 9 open reading frame gene
*FUS*: Fused in sarcoma gene
IBMPFD: Inclusion body myopathy associated with Paget disease of bone and frontotemporal dementia
*MATR3*: Matrin 3 gene
MATR3: Matrin 3 protein
MM: Mild to moderate phenotype
MoPrP: Mouse prion promoter
NMJ: Neuromuscular junction
NT: Non-transgenic
PBS: Phosphate buffered saline
S: Severe phenotype
*SOD1*: Superoxide dismutase I gene
*TARDBP*: Tar-DNA binding protein gene
TBS: Tris-buffered saline
TDP-43: TAR DNA binding protein 43
Tg: Transgenic
UTR: Untranslated region
VCP: Valosin containing protein
*VCP*: Valosin containing protein gene
ZNP1: Synaptotagmin 2
